The article "Service Migration Policy Optimization considering User Mobility for E-Healthcare Applications" was published in 2021. Journal: J Healthc Eng.

# Service Migration Policy Optimization considering User Mobility for E-Healthcare Applications

**DOI:** 10.1155/2021/9922876

**Published:** 2021-06-19

**Authors:** Xuhui Zhao, Jianghui Liu, Baofeng Ji, Lin Wang

**Affiliations:** Information Engineering College, Henan University of Science and Technology, Luoyang 471000, China

## Abstract

Mobile edge computing (MEC) is an emerging technology that provides cloud services at the edge of network to enable latency-critical and resource-intensive E-healthcare applications. User mobility is common in MEC. User mobility can result in an interruption of ongoing edge services and a dramatic drop in quality of service. Service migration has a great potential to address the issues and brings inevitable cost for the system. In this paper, we propose a service migration solution based on migration zone and formulate service migration cost with a comprehensive model that captures the key challenges. Then, we formulate service migration problem into Markov decision process to obtain optimal service migration policies that decide where to migrate in a limited area. We propose three algorithms to resolve the optimization problem given by the formulated model. Finally, we demonstrate the performance of our proposed algorithms by carrying out extensive experiments. We show that the proposed service migration approach reduces the total cost by up to 3 times compared to no migration and outperforms the general solution in terms of the total expected reward.

## 1. Introduction

With the development of Internet of Things, E-healthcare applications are emerging and gaining popularity. These E-healthcare applications require low latency and intensive resource (computation or storage resource). However, IoT terminals (sensors or vehicles) have limited resources (low processing speed, small storage capacity, and limited battery life), which is insufficient to complete these applications. To mitigate this limitation, mobile edge computing (MEC) is envisioned as a promising paradigm by providing cloud service at the edge of network [1, 2]. By leveraging cloud service deployed near mobile terminals, the latency of IoT applications can be significantly guaranteed and the quality of experience of mobile user can be greatly improved. Suppose a patient travelling in a vehicle needs monitoring the health parameters continuously such as blood pressure and pulse rate, which are collected by IoT devices and the raw health data are sent to the edge service site through the client E-healthcare application. The edge site processes the data based on the predeployed E-healthcare application and sends the processed result to the client application. Thus, MEC is assumed a key enabling technology for realizing the E-healthcare visions.

User mobility is common in MEC systems. The edge sites often place cloud resources on the edge access devices such as base stations (BSs) in cellular system and access points (AP) in Wi-Fi. Network virtualization allows heterogeneous networks to coexist on a shared infrastructure, and, hence, it can be considered as a solution for the heterogeneity in MEC [3, 4]. On the other hand, user mobility can result in interruption of ongoing edge services and dramatic drop in QoS, and service migration (SM) has a great potential to address the issues [5, 6]. SM policy should be made such that whether and where to migrate the ongoing edge services as an arbitrary user moves outside the service area of the associated edge cloud site, which involves multiple challenges: first, a user may connect to one edge cloud in one time slot and switch to another in the next. Consequently, communication resources (bandwidth) and computing resources (virtual machine size) may be reconfigured in each time slot, which incur reconfiguration cost due to heterogeneity in edge cloud. Second, it is hard to predict how each user will move over time in some scenarios, especially in vehicle networks. Under the circumstances with no assumption about user mobility, migration policy still needs to be made in order to ensure service continuity. Third, from the perspective of communication resources, it is most advantageous to migrate the cloud service to the location closest to the user; however, from the perspective of computing resources, this approach has been demonstrated to be inadequate due to the dynamic workloads of the network [7–9].

Despite the extensive existing research on mobility-induced service migration in the edge cloud context in general, fine grained and random mobility features are not considered [5, 8–10], and most of them often assume prior knowledge about user mobility [11–14]. In addition, migration policy design in the research only considers whether and where to migrate. And edge cloud service is always migrated to the cloud server closest to the user. When mobile users have multiple access edge clouds, where to migrate should be considered extensively in terms of fine-grained mobility. The transmission cost and migration cost have been well considered in the existing research; nevertheless, none of them considers the influence of user mobility on reconfiguration induced by service migration.

Based on the above observations, we study the user-mobility-driven optimization of the resource usage, reconfiguration, and migration altogether in edge clouds without mobility model assumption. We use the MDP framework to study service migration jointly considering user mobility and heterogeneity in edge clouds. We make three contributions:

1. Our formulation captures multiple types of important costs. The first is resource usage cost associated with service location depending on resource price strategy for the MEC system. The second is the reconfiguration cost accounts for changes in resources. Network reconfiguration in virtualization incurs a cost for the system by remapping a subset of virtual nodes or links to better align the allocation of resources to current network conditions. The third is migration time cost for guaranteeing quality of service. We pursue the optimization of the total cost while serving each user's workload from the perspective of edge cloud operator.
2. We provide a mathematical framework to design optimal service migration policies that decide where to migrate without assumption of user mobility in a limited area. We formulate service migration problem into Markov decision process (MDP). We propose Service Migration algorithm based on Value Iteration (SMVI), In-place Value Iteration (SMIVI), and Policy Iteration (SMPI) to resolve the optimization problem given by the above cost model.
3. We demonstrate the performance of our proposed algorithms by carrying out extensive experiments. We compare the proposed policy with several baseline strategies that include no migration, migration without considering reconfiguration cost. It is shown that the proposed approach offers significant gains over those baseline approaches. The results show that, up to 3 times compared to no migration, up to 5% reduction on the total cost can be achieved compared to the approaches typically employed in edge clouds.

The remainder of the paper is organized as follows. In the next section, we review some related service migration in MEC and their problems. In Section 3, we describe the system model and the basic assumptions considered in this paper. Then, we formulate the problem of designing an optimal service migration policy as MDP. We detail the proposed algorithm in Section 4. To validate the proposed study, we provide numerical experiments under various settings in Section 5. Finally, we draw the conclusions in Section 6.

## 2. Related Work

Induced-mobility service migration has been paid much attention in MEC system. The related research work contains optimization of migration policy and execution of migration.

### 2.1. Optimization of Migration Policies

Migration can bring benefits and incur computation and communication resource overheads. Therefore, the decision on whether and where to migrate depends on many aspects, such as user mobility, the number of simultaneous migrations, resource availability at heterogeneous edge clouds, and so on, which is a sophisticated optimization problem. The study in [8] aimed to optimize service migration policy aiming at avoiding the migration if the stable delay is acceptable. They assumed that a required end-to-end latency threshold is known in advance. Meanwhile, they do not consider the workloads of destination edge cloud as well as their reconfiguration costs for the service. The study in [9] proposed a service migration policy to decide the services that are run on the mobile edge nodes to be migrated. This problem is solved by a Lyapunov-based approach. The optimal migration strategy is obtained in closed form, and an online algorithm outputs the number of service replicas (how many) and where these services are to be migrated prior to the handover execution. The proposed mathematical models are based on simple assumptions and thus cannot cope with complex mobility condition and user context information. The authors of [5, 11, 12] studied service migration design under the one-dimensional and two-dimensional mobility model, and the study in [11] proposed stochastic frameworks for dynamic workload migration based on the Lyapunov optimization technique. And references [5, 12] also did not consider the reconfiguration costs for the service, which cannot be directly used in heterogeneity in edge cloud network. Although the study in [11] considered the reconfiguration cost in the problem formulation, it is only assumed that the reconfiguration cost is the function of distance. However, the parameter in the formulation was not easy to determine in practice. In addition, all of them either require statistics information or model on user mobility.

The realization of cloud service depends on virtualization technology represented by virtual machine (VM). The authors of [15] proposed strategies to find suitable bandwidth and precopy iteration count to optimize different performance metrics of VM migration over a WAN. The formulated models were to optimize network resource consumption, migration duration. And a strategy was proposed to determine appropriate the migration bandwidth and number of precopy iterations, and it performed numerical experiments with large number of migration requests. The authors of [16] studied the problem of optimal VM placement and migration to minimize resource usage and power consumption in a data centre. The formulated problem was optimized as a joint multiple objective function and solved by leveraging the framework of convex optimization. A multilevel join VM placement and migration algorithms provided an approximate optimal solution. However, the above work considered the centralized cloud environment instead of edge clouds. In the edge cloud environment, mobile terminals are diversified, and the mobility of different mobile terminals is more complex and has a certain degree of randomness.

Our model captures multiple types of important costs. The first is transmission cost, depending on service location. Edge cloud is usually collocated with an access point (AP, a cellular base station, or a Wi-Fi access point); therefore, different cloud resources may have different prices controlled by resources price strategy for the MEC system [17]. The second is the reconfiguration cost accounts for changes in resources. Although network virtualization is considered as the most promising approach to realize heterogeneous networks to coexist on a shared infrastructure, network reconfiguration in virtualization incurs a cost for the system by remapping a subset of virtual nodes or links to better align the allocation of resources to current network conditions [18]. This reconfiguration cost cannot be neglected to improve the total net gain for the edge cloud service provider [3]. The third is migration time cost. Specifically, the factors affecting VM migration time are the memory size, the number of concurrent VM on destination server, and the available network bandwidth [19]. Without any knowledge on user mobility, our algorithm makes optimal migration decisions while guaranteeing system reward.

### 2.2. Execution of Migration

Execution of migration focuses on how to efficiently execute live migration in a practical MEC system. The framework proposed in [20] aimed at smooth migration of all or only a required portion of an ongoing IP service between a data centre and user equipment. The service migration and continuity were supported by replacing IP addressing with service identification. Recent efforts toward the implementation of service migration in MEC environments have focused on VM migration [21–25]. The study in [21] proposed a technique that initiates the migration of VMs between heterogeneous cloud environments. The author demonstrates heterogeneous VM migration between various cloud platforms built on different architectures. The study in [22] presented a three-layer framework for migrating active service applications that are encapsulated either in VMs or in containers. It aims at maintaining relatively low service downtime and overall migration time. Especially, the framework applied to both virtual machines and containers. The authors of [23] proposed Follow Me Fog, a framework supporting a new seamless handover timing scheme among different computation access points by designing a job premigration mechanism. The authors of [24] proposed remote loading and redirection to accelerate the service migration. By tracing historic access patterns, the proposed method first generates a loading request list that locates the core codes in the image file of service applications for booting. The study in [25] gave an overview of VM migration and discussed both its benefits and challenges, the studies regarding linking VM migration to user mobility are summarized as well, and further optimizations on live VM migration were listed in the paper. In conclusion, the above research provides a solid research foundation for the implementation of service migration strategy proposed in this paper.

## 3. Model Formulation

Considering the scenario as shown in Figure 1, an edge server contains one or more physical machines hosting several VMs, covering the mobile users in proximity. These edge servers are interconnected with each other via different kinds of network connections supported by network virtualization reconfiguration [3, 18].

Note that we use edge server or edge cloud site as a general term. In our system model, there are N edge servers that are virtualized and managed by a SM Management Entity (SMME). The edge cloud pointed by red or green arrows denotes the available access edge clouds, and the black one-way arrow indicated the ambulance moved from the current position to another position.

Migration policy is triggered whenever an ambulance is in its migration zone in an access point, as shown in Figure 2. SMME should decide which edge cloud to migrate when mobile users have multiple access edge clouds. In this work, this zone is determined based on a fixed distance to the AP or dynamic distances based on the user's speed and VM size. We assume that the ambulance moves around in a limited area in the city.

We utilize access point A and MEC-A as the source edge site and access point B and MEC-B as the destination edge site. Handover management entity (HME) is used to implement handover policy and handover procedure. The whole mechanism of service migration can be described as follows, which is shown in Figure 3.

  Step 1: a patient travelling in a vehicle accesses the E-healthcare application hosted by MEC-A.
  Step 2: the access point A sends the position information of the related vehicle to the handover management entity.
  Step 3: when the vehicle enters the migration zone of an access point, the HME implements handover procedure and informs the SMME to make a decision about service migration.
  Step 4: the SMME implements service migration policy by our proposed approach, the result of implementing our algorithm is supposed as MEC-B, and then the SMME informs the MEC-A to implement service migration procedure.
  Step 5: the service migration is implemented between MEC-A and MEC-C.
  Step 6: the vehicle enters the coverage of access point B.
  Step 7: the E-healthcare application service is resumed in the MEC-B.
  Step 8: the service migration is completed.
  Step 9: all the resources are released including bandwidth, storage, and computation resources hosted by MEC-A and MEC-B.

In the following sections, we describe our model for each component in an edge cloud system; then, we formulate the service migration problem.

### 3.1. Edge Cloud System

We consider an edge cloud system (e.g., *N*=5 × 5) where a vehicle accesses a cloud-based service hosted on the MECs. The set of possible edge cloud locations is given by *l*=(*i*, *j*),  *l* ∈ *L*, where *L* is assumed to be finite. An edge cloud is defined as a pool of virtualized computing resources, which is usually collocated with a cellular base station, a Wi-Fi access point, or Mobile Cloudlets. The maximum workload of an edge cloud *l* is defined as *c*_*i*,*j*_. These edge servers are interconnected with each other. The network bandwidth between two edge clouds *l* and *l*′ is given by *B*(*l*, *l*′). The number of concurrent running workloads of all the edge clouds is denoted by the set *W*={*w*_*ij*_}, ∀(*i*, *j*) ∈ *L*.

### 3.2. Mobile Terminals' Mobility and Migration

We assume an ambulance *u* (also called mobile terminal) with IoT devices move around in the limited area that is shown as grids in Figure 2. In a certain time slot, the ambulance connects to an edge cloud *l* ∈ *L* that covers the vicinity of the ambulance and accesses the E-healthcare application service, incurring an allocated bandwidth *x*_*u*_ and the number of CPU processing cycles *m*_*u*_, and the corresponding virtual machine state data size is denoted by *d*_*u*_. When the ambulance leaves the limited coverage of the current edge cloud, the corresponding cloud service can be migrated to one of the available neighbour edge clouds for the purpose of cloud service continuity. As shown in Figure 4, the cloud service at the edge of the grid can migrate to the surrounding two neighbour clouds, while the cloud service at other locations plotted by red line can be migrated to the surrounding four neighbours. For example, edge cloud services in the location of edge cloud (0, 0) can be migrated to (0, 1) or (1, 0). As another example, services in the edge cloud (2, 2) can be migrated to (1, 2), (3, 2), (2, 1), or (2, 3). SM management entity should decide which edge cloud to migrate as an ambulance moves around in the limited area.

### 3.3. Costs

We consider three aspects of costs in the edge cloud system: the edge cloud usage cost, the migration cost, and the reconfiguration cost. These costs are able to represent the most prominent expenditure from the perspective of the cloud operator.

#### 3.3.1. Resource Usage Cost

In this paper, we assume that the resource usage cost refers to bandwidth incurring by data transmission and computation resources usage incurring by task processing, which can be expressed as

(1) $$\begin{array}{c} \text{Cos}t_{\text{usa}}=a_{l}*x^{t}+b_{l}*\frac{m^{t}}{100}, \end{array}$$

where _*x*_^*t*^ denotes the bandwidth at current location *l* at time slot *t*, *x*^*t*^ < *λ*_*u*_ and *a*_*l*_ denotes the unit cost of bandwidth resource at location *l*. *m*^*t*^ measures the number of CPU processing cycles at time slot *t*. *b*_*l*_ represents the cost of using 100 MHz CPU.

#### 3.3.2. Reconfiguration Cost

As an ambulance move around in the limited area, the SMME may migrate the workload from source edge cloud to destination edge cloud decided by migration policy, which results in adapting the amount of resources allocated in destination edge cloud. Such adaptation depends on the number of reallocated virtual links and nodes, which would incur some inevitable cost for preparing the resources. The reconfiguration cost of allocating 100 MHz CPU and 1 Mbps bandwidth is denoted by *p*_*l*_ for edge cloud *l*; the reconfiguration cost is calculated as

(2) $$\begin{array}{c} \mathrm{Cos}\;t_{\text{rec}}=p_{l}\left[\left(x^{t}-x^{t-1}\right)+\frac{\left(m^{t}-m^{t-1}\right)}{100}\right]. \end{array}$$

#### 3.3.3. Migration Cost

This cost represents the delay when we migrate the workload from one edge cloud to another due to data movement. Specifically, the major factors impacting VM migration time are the memory size, memory dirtying rate of the VM to be migrated, and the available network bandwidth, as well as the number of concurrent running VM at the destination server [16]. For simplicity, we approximately calculate the migration time as

(3) $$\begin{array}{c} \text{Cos}t_{\text{mig}}=d_{u}^{t}*\frac{w_{l^{\prime }}}{B_{l,l^{\prime }}}, \end{array}$$

where *d*_*u*_^*t*^ denotes the virtual machine's data size at time slot *t*, *w*_*l*′_ denotes the number of concurrent running VM in destination cloud *l*′, and *B*_*l*,*l*′_ denotes network bandwidth between edge cloud *l* and *l*′.

### 3.4. Problem Formulation

By combining the essential models above, we formulate the migration policy as MDP. In order to obtain the optimal policy, it is necessary to identify the actions, state, and reward functions in our mathematical model, which is given in the following sections.

#### 3.4.1. System State

Let *S*^*t*^ denote the system state at time *t*, defined by (*l*^*t*^, *o*^*t*^), where *l*^*t*^ is the locations set of cloud service at time *t*, and *o*^*t*^ denotes the workloads at the current location *l*^*t*^, where *o*^*t*^=(*x*_*u*_^*t*^, *m*_*u*_^*t*^, *d*_*u*_^*t*^). Consequently, the state vector can be described as *S*^*t*^=(*l*^*t*^, *o*^*t*^). Here, *l*^*t*^=(*i*, *j*), for ∀*i* < *N*,  *j* < *N*.

#### 3.4.2. System Action

In the system, the SMME decides where to migrate the edge cloud service when a vehicle moves around in the limited area. It is not optimal to migrate the service to a location that is farther away from the user, as one would intuitively expect. Therefore, we assume that when the vehicle is in the migration zone in the current edge cloud, the corresponding cloud service can be migrated to one of the available neighbour edge clouds. The current action is represented by *a*, *a* ∈ *A*, *A*={0,1,2,3}, where 0 represents migration to the north, 1 represents migration to the south, 2 represents migration to the west, and 3 represents migration to the east.

#### 3.4.3. Reward Function

Our goal is to design a policy that uses the E-healthcare application's workload (bandwidth, or CPU consumption) and service location as input, and the policy continuously decides where to migrate the workload for each vehicle as it moves, such that the total cost is minimized over time. Note that the reward function in MDP is the maximum value; we set three mapping variables Cos  *t*_usa_′, Cos  *t*_mig_′, and Cos  *t*_rec_′, corresponding to the three original variables. Therefore, the reward function is the weighted sum of the resource usage cost, migration cost, and reconfiguration cost, as given by

(4) $$\begin{array}{c} C^{t}=\alpha *\;\mathrm{Cos}\;t_{\text{usa}}^{\prime }+\beta *\;\mathrm{Cos}\;t_{\text{rec}}^{\prime }+\chi *\;\mathrm{Cos}\;t_{\text{mig}}^{\prime }, \end{array}$$

where *α*, *β*, and *χ* are the weights of the three types of cost, respectively. Cos  *t*_*usa*_′, Cos  *t*_mig_′, Cos  *t*_rec_′ denotes the corresponding cost after being normalized, and min () and max () are minimum and maximum functions of a variable.

(5) $$\begin{array}{c} \mathrm{Cos}\;t_{\text{usa}}^{\prime }=1-\frac{\cos\;t_{\text{usa}}-\min\left(\cos\;t_{\text{usa}}\right)}{\max\left(\cos\;t_{\text{usa}}\right)-\min\left(\cos\;t_{\text{usa}}\right)},\\ \mathrm{Cos}\;t_{\text{rec}}^{\prime }=1-\frac{\cos\;t_{\text{rec}}-\min\left(\cos\;t_{\text{rec}}\right)}{\max\left(\cos\;t_{\text{rec}}\right)-\min\left(\cos\;t_{\text{rec}}\right)},\\ \mathrm{Cos}\;t_{\text{mig}}^{\prime }=1-\frac{\cos\;t_{\text{mig}}-\min\left(\cos\;t_{\text{mig}}\right)}{\max\left(\cos\;t_{\text{mig}}\right)-\min\left(\cos\;t_{\text{mig}}\right)}. \end{array}$$

Take expectation with respect to service migration costs in each epoch over the randomized network states *S*^*t*^ and the actions *A*^*t*^ induced by a given control policy *π*. This action causes the system to transition to a new intermediate state *S*^*t*+1^=(*l*^*t*+1^, *o*^*t*+1^). The expected long-term reward of the MEC conditioned on an initial network state *S*^1^ can be expressed as

(6) $$\begin{array}{c} V\left(S,\pi \right)=E_{\pi }\left[\left(1-\gamma \right)\sum_{t=1}^{\infty }{\left(\gamma \right)}^{t-1}C^{t}|S^{1}=S\right], \end{array}$$

where *γ* ∈ [0,1) is the discount factor and (*γ*)^*t*−1^ denotes the discount factor to the (t − 1)-th power. The objective of the MEC system is to design an optimal control policy *π*^*∗*^ that maximizes *V*(*S*, *π*), for any given initial network state S, which can be formally formulated as

(7) $$\begin{array}{c} \pi^{*}=\underset{\pi }{\arg}\max V\left(S,\pi \right). \end{array}$$

We denote *V*(*S*)=*V*(*S*, *π*^*∗*^) as the optimal state-value function.

## 4. Solving the Optimal Control Policy

Note that standard approaches of solving for the optimal policy of an MDP include value iteration and policy iteration [26]. To derive the service migration policy, we propose SMVI and SMPI algorithm, respectively. The details can be described as follows.

The SMPI algorithm (Algorithm 1) contains two parts: policy evaluation (Algorithm 2) and policy improvement (Algorithm 3). Firstly, the V-function and the policy are initialized randomly. Then, for the current policy, the value function of the state *s* under the policy is estimated by the algorithm of iterative policy evaluation, and a new strategy is obtained by greedy policy improvement. The above procedure is looped until the policy remains unchanged. The pseudo codes of the algorithms are as follows:

In order to find the optimal strategy, the SMVI algorithm (Algorithm 4) uses the Bellman optimal equation to iterate. However, there is no explicit strategy in the update process, so the value function in the iteration process may not correspond to any strategy. Additionally, we propose service migration algorithm based on the In-place Value Iterative (SMIVI); the difference between the in-place value iterative method and the general value iterative method is asynchronous update in the algorithm. That is to say, the V update is directly performed during the update process. The marked line with 16 in Algorithm 4 is replaced by sentence *V* [*i*, *j*] = *np*.max (*qs*), which generate the SMIVI algorithm. The pseudo code of SMVI algorithm is as follows:

### 4.1. Evaluation

The number of actions in MDP formulated by service migration problem is four, because the edge cloud service can only be migrated to the four available neighbour edge clouds. The variable *N*_action is assumed as a constant in all the algorithms. Therefore, the execution time of all the algorithms depends on the execution times implemented by the body code of “for” loop, the time complexity of Algorithm 1, Algorithm 2, Algorithm 3, Algorithm 4 are O(n), O(n^2^), O(n), O(n^2^), respectively.

We validate the performance of the proposed service migration algorithm based MDP in Python. We use PyCharm as the Python integrated development environment. All the experiments are implemented on a computer with Intel Core i5-4200U CPU 2.3 GHz and 4096 MB RAM. We conduct extensive experiments and report the experimental results in this section. In addition to the proposed algorithm, other schemes are taken as the performance reference for comparison on the same topology with the same parameter setting, which are described as follows.

#### 4.1.1. No Migration

No matter how the vehicle moves, the system will not take the migration action.

#### 4.1.2. Other Schemes [5, 12]

The migration policy does not consider the reconfiguration cost.

All the measurements were performed on a computer equipped with Intel Core i5-6500 CPU (3.2 GHz) and 8.0 GB RAM.

## 5. Experimental Settings

We consider an edge cloud system deployed with 25 edge clouds, as shown in the grid of Figure 2; the allocated bandwidth at different locations follows uniform distributions over (4, 100). The available network bandwidth between the source and destination edge servers was between 20 and 100 MBps. The number of concurrent running VM in each edge cloud server follows random distribution over (1, 25). The VM size was between 800 MB and 1700 MB [27]. The reconfiguration price varies among different edge clouds. We generate the reconfiguration prices following a Gauss distribution with the mean 20-euro and the standard deviation 5-euro. We categorize all the edge clouds into three clusters, each of which is subscribed to one of three bandwidth prices provided by Internet providers. The average prices are 2.49 euro/Mbps, 4.86 euro/Mbps, and 1.25 euro/Mbps, respectively [28].

### 5.1. The Optimal Migration Policy under Different Scenarios

As mentioned before *α*, *β*, and *ω* denote the weights of the three types of cost, respectively. Three parameter settings are envisioned:

1. *α*=0.8, *β*=0.1, and *χ*=0.1 which represents a high resource usage cost compared to migration cost and reconfigure cost if a service migration is launched.
2. *α*=0.1, *β*=0.8, and *χ*=0.1 which represents a high migration time cost compared to resource usage cost and reconfigure cost if a service migration is launched.
3. *α*=0.1, *β*=0.1, and *χ*=0.8 which represents a reconfiguration cost compared to resource usage cost and migration cost if a service migration is launched.

Figures 5–7 illustrate the optimal policy constructions for the three above-mentioned settings. Arrows in the figure indicate the optimal migration direction. For instance, when *α*=0.1, *β*=0.1, *χ*=0.8, the optimal policy recommends service in the location (0, 0) migrating to the east-(0, 1). However, when *α*=0.1, *β*=0.8, *χ*=0.1, the optimal policy recommends the same service migrating to the south-(1, 0). This is because reconfiguration cost incurring by migration to the location (0, 1) is greater than that of location (1, 0). The optimal policy recommends migration to the south for increasing total reward. Note that the weight parameters have a great impact on the optimal policy construction, since migration to different location incurs different migration cost and reconfiguration cost. This difference is not negligible in comparison to the achieved gain when migrating a service.

### 5.2. Impact of Weights of the Three Costs on the Expected Reward

We report also in Figure 8 the impact of the parameter's weights of the three costs on the total expected reward by varying its value in three cases:

  Case 1: *α* takes a fixed value 0.1, *β* progressively increases from 0.1 to 0.8, and *χ* progressively decreases from 0.8 to 0.1
  Case 2: *β* takes a fixed value 0.1, *α* progressively increases from 0.1 to 0.8, and *χ* progressively decreases from 0.8 to 0.1
  Case 3: *χ* takes a fixed value 0.1, *α* progressively increases from 0.1 to 0.8, and *β* progressively decreases from 0.8 to 0.1

It is notable that the maximum reward that each algorithm can achieve may be different when parameters take different values; i.e., the maximum expected reward over *α*=0.1, *β*=0.1, *χ*=0.8 is 9.012, which is the same as parameter settings over *α*=0.8, *β*=0.1, *χ*=0.1. However, the maximum expected reward over *α*=0.1, *β*=0.8, *χ*=0.1 can only reach 6.8, which is smaller than that of the other two parameter settings.

We observe that when *α* takes a fixed value 0.1, the expected system reward progressively decreases. This is because reconfiguration cost and migration cost dominate more system cost. While *χ* takes a fixed value 0.1, the expected system reward progressively increases. This is because increment of weights of resource usage cost can bring more reward under our system context parameter settings. It is notable that with the increase of *α*, the expected reward of our algorithm declines slightly at the beginning and then increases to a stable level when *β* takes a fixed value 0.1. And the expected reward over *α*=0.1, *β*=0.1, *χ*=0.8 can reach the maximum value 9.012.

### 5.3. Comparison of the Convergence Speed of Different Algorithms

In this section, we compare the convergence speed of different algorithms. Here are two settings to be considered.

#### 5.3.1. Total Expected Reward versus the Number of Iteration Update Steps

From Figures 9–11, we observe that our algorithm performs in a similar way under different parameter settings. We can see that when update step takes the same value, the convergence speed of policy iteration algorithm is the fastest and value iteration is the slowest. This is because value iteration finds the optimal policy from the Bellman's equation iteratively, which may require many iterations before converging to the optimal result. Policy iteration generally requires a smaller number of iterations. Moreover, SMPI finds the exact values of the discounted sum cost for the policy resulting from the previous iteration. SMPI converges at about 7 iterations, while SMVI and SMIVI converge until almost 40 iterations and maintain steady performance thereafter.

#### 5.3.2. Total Expected Reward versus Update Time

As shown in Figures 12 and 13, when update time takes the same value, the convergence speed of SMIVI is faster than other algorithms, and SMPI is the slowest (SMVI and SMIVI algorithm converge until almost 0.02 seconds while SMPI algorithm converges at about 5 seconds). This is because SMPI algorithm uses greedy method to improve policy, while the greedy policy improvement generates a lower efficiency.

### 5.4. Performance Comparison with Other Migration Policies

In this section, we compare the Proposed Migration Policy considering three costs (PMP) with two benchmark methods in the experiments: the migration strategy only considers Resource Usage cost and Migration Cost strategy (RUMC) [3, 10] and no migration. All the experiments are implemented under the parameter settings with *α*=0.8, *β*=0.1, *χ*=0.1.

It must be noted that the factors considered by different algorithms are not the same, it is difficult to compare directly. For the policy that considers only the communication cost and the migration cost, we first make the corresponding migration decision through the flow of the policy itself and then calculate the reward of this action in the current state according to the function defined in this paper. From the results shown by Figures 14–16, we can see that our PMP implemented by all the three algorithms (SMPI, SMVI, and SMIVI) performs better than RUMC and no migration. That is because RUMC always choosees the destination location that generates the minimum transmission cost and migration cost, while PMP may select one of the four neighbours edge servers as destination considering the reconfiguration cost at the destination location. Compared to no migration, PMP can increase reward by three times. Compared to RUMC, PMP can increase reward by 5%.

## 6. Conclusion

In this paper, we design a service migration policy considering mobile terminal's mobility and heterogeneity in edge cloud systems. Our formulation captures general cost models involving transmission cost, migration cost, and reconfiguration cost. We provide a mathematical framework to design optimal service migration policies that decide where to migrate without assumption of mobile terminal's mobility model in a limited area; namely, the policy triggers service migration each time a mobile terminal enters migration zone. We formulate service migration problem into MDP. Value iteration and policy iteration algorithms are used to resolve the optimization problem given by the formulized model. The SMME can optimally decide where a service needs to be migrated. The performance of the main algorithms is demonstrated by extensive experiments. The results show that the proposed service migration mechanism always achieves the maximum expected reward compared to two other policies. The proposed method is suitable for the service migration in limited area. For the large-scale networked MEC systems, the huge state space will lead to the performance degradation of the algorithms. In the future work, we will study live migration method and performance under large-scale networked MEC systems.

## Figures and Tables

**Figure 1:** A case of service migration in mobile edge computing. The edge cloud pointed by red or green arrows denotes the available access edge clouds, and the black one-way arrow indicates that the ambulance moved from the current position to another.

**Figure 2:** Migration zone.

**Figure 3:** The whole mechanism of service migration.

**Figure 4:** Mobile terminals move around in a limited area.

**Figure 5:** The optimal policy constructed by SMPI over *α*=0.1, *β*=0.1, and *χ*=0.8.

**Figure 6:** The optimal policy constructed by SMPI over *α*=0.1, *β*=0.8, and *χ*=0.1.

**Figure 7:** The optimal policy constructed by SMPI algorithm over *α*=0.8, and *β*=0.1, *χ*=0.1.

**Figure 8:** The impact of the parameter's weights of the three costs on the total expected reward.

**Figure 9:** The expected reward over *α*=0.1, *β*=0.1, and *χ*=0.8.

**Figure 10:** The expected reward over *α*=0.1, *β*=0.8, and *χ*=0.1.

**Figure 11:** The expected reward over *α*=0.8, *β*=0.1, and *χ*=0.1.

**Figure 12:** The expected reward versus times, implemented by SMPI algorithm with *α*=0.8, *β*=0.1, and *χ*=0.1.

**Figure 13:** The expected reward versus times, implemented by SMVI and SMIVI with *α*=0.8, *β*=0.1, and *χ*=0.1.

**Figure 14:** The results of implementing SMPI.

**Figure 15:** The results of implementing SMVI.

**Figure 16:** The results of implementing SMIVI.

**Algorithm 1:** SMPI (policy, env, max_step = 100, tol = 1e-6).

**Algorithm 2:** Value_evaluate (policy, env, max_step = 100, tol = 1e-6).

**Algorithm 3:** Policy_improvement (env, *V*).

**Algorithm 4:** SMVI (max_iter = 100, max_step = 100, tol = 1e-6).

## Data Availability

The data used to support the findings of this study are available from the corresponding author upon request.
